# Analgesic, Anti-inflammatory, Antipyretic, and *In Silico* Measurements of *Sonneratia caseolaris* (L.) Fruits from Sundarbans, Bangladesh

**DOI:** 10.1155/2022/1405821

**Published:** 2022-08-24

**Authors:** Pritam Kundu, Shovan Lal Debnath, Hiron Saraj Devnath, Lopa Saha, Samir Kumar Sadhu

**Affiliations:** Pharmacy Discipline, Life Science School, Khulna University, Khulna 9208, Bangladesh

## Abstract

*Sonneratia caseolaris* is a widely distributed mangrove plant having much therapeutic importance in traditional medicine. This plant is reported for possessing numerous compounds that are already used for many therapeutic purposes. After finding the presence of antioxidant components in the qualitative antioxidative assay, we went to conduct quantitative tests where the total contents of phenolics, flavonoids, and tannins were estimated as 122 mg GAE/gm, 613 mg QE/gm, and 30 mg GAE/gm, respectively. In DPPH free radical, H_2_O_2_, and superoxide radical scavenging assay, the SC_50_ values were found to be 87, 66, and 192 *μ*g/ml, respectively. In FeCl_3_ reducing power assay, the RC_50_ of SC extract and ascorbic acid were 80 and 28 *μ*g/ml, respectively. This extract revealed a significant peripheral analgesic effect in the acetic acid-induced writhing model in mice by reducing the writhing impulse by about 21% and 39% at 250  and 500 mg/kg doses, respectively, and a central analgesic effect in the tail immersion method by elongating the time up to about 22% and 37% at the same doses. In the anti-inflammatory test in mice, this extract reduced the paw edema size over the observed period in a dose-dependent manner. It also showed a significant reduction in the elevated rectal temperature of mice in the observing period in Brewer's yeast-induced pyrexia model. *In silico* analysis revealed better binding characteristics of ellagic acid and luteolin among other compounds with various receptors that might be responsible for antioxidative and anti-inflammatory properties. From our observation, we suppose that SC fruits might be a potential source of drug leads for various inflammatory disorders.

## 1. Introduction

Plants possessing valuable characteristics which assure them as drugs and can be used for therapeutic purposes are known as medicinal plants. Nature has always blessed us with its numerous medicinal plants to get remedies for many diseases from the very ancient age. Although there has been much development in different modern technologies such as combinatorial chemistry, bioinformatics, and computer-aided drug design, still, medicinal plants provide approximately half of the medicines currently in clinical use [1]. In this project, we performed both qualitative and quantitative antioxidative tests. We evaluated peripheral analgesic activity by the acetic acid-induced writhing method which is a well-recognized method of determining analgesic effect. On the other hand, central analgesic activity was evaluated by the tail immersion method which can measure the elongation of tail immersion time that is directly linked with the central nervous system pain management. Anti-inflammatory activity was determined by the formalin-induced paw edema method where reduction of edema size over the observing period directly denotes the degree of inflammation. By Brewer's yeast-induced pyrexia method, the antipyretic effect was evaluated where lowering of the rectal temperature indicated the antipyretic property. After these experiments, *in silico* analysis of six antioxidant molecules present in this extract with different proteins revealed the binding characteristics and justified our experimental results.

*Sonneratia caseolaris* (Cork tree) is an evergreen mangrove tree belonging to the family Sonneratiaceae (Figure 1). This plant is widely found in the mangrove forests of different countries of the world such as India, Sri Lanka, China, Cambodia, Thailand, Vietnam, Indonesia, Malaysia, Philippines, northern Australia, and the Pacific Islands. In Bangladesh, this plant (locally named Choila, Ora) is widely available in the tidal forests of Barisal, Chattogram, Chokoria, and Sundarbans. This much-branched tall (up to 15 m) tree has underground roots and pneumatophores (breathing roots). Its flowers are dark red petalled. The green fruits are spherical, about 5-7.5 cm wide. Barks are grey and coarsely flaky [2, 3]. Upon reviewing different articles, several compounds have been found to be present in this plant. Wu et al. isolated oleanolic acid, *β*-sitosterol-*β*-D-glucopyranoside, (–)-*R*-nyasol, (–)-*R-*4′*-*O*-*methylnyasol, luteolin, luteolin 7-O-*β*-glucoside, and maslinic acid from its fruits, whereas Dev et al. reported the presence of ellagic acid, vanillic acid, and myricetin upon HPLC analysis [3, 4]. Sadhu et al. isolated two flavonoids, namely, luteolin and luteolin 7-O-*β*-glucoside from SC leaves, whereas Wetwitayaklung et al. confirmed the presence of maslinic acid, sterols, and triterpenoids [5, 6].

This plant has tremendous importance in the folklore medicine system. The ripened fruits of SC have an appealing flavor and taste, enriched with vitamins. People of Bangladesh cook condiments from its fruits and use the fruits to treat toothache, swelling, bleeding disorders, and as an antiseptic. Malayan and Thai people use it as an expectorant, emollient, anthelmintic, and blood coagulant [6, 7]. Compounds reported from various parts of this plant are already well recognized for eliciting different types of biological benefits. Proper investigation of different parts of this plant may signify its traditional usage in a scientific manner. However, most of the reported scientific works were carried out on its leaves and bark. Considering the traditional usage of its fruits for pain and swelling management and the presence of numerous valuable constituents in fruits, we aimed our focus to assess the antioxidative, analgesic, anti-inflammatory, and antipyretic properties. Then, *in silico* analysis was also carried out to determine the proper binding characteristics of the compounds (ligands) with specific receptors (proteins) in our body.

## 2. Materials and Methods

### 2.1. Schematic Overview of the Experimental Program

Figure 2 represents a schematic diagram of this experimental program. After the collection of *S. caseolaris* fruits from Mongla, Bagerhat, in 2017, the dried plant sample was identified by the experts in Bangladesh National Herbarium (DACB-43821); cold extraction with 96% ethanol for 15 days was carried out to obtain the crude extract with 3.3% *w*/*w* yield; after the procurement of Swiss albino mice (4-5 weeks old, average body weight 20-25 gm) from the animal house of Jahangirnagar University, those were got adapted in the animal house of Khulna University to conduct the pharmacological tests.

This work was directed to establish the scientific basis of the traditional usage of *S. caseolaris* fruits.

In order to conduct the pharmacological experiments in mice with the proper ethical standard and guidelines, approval from the Animal Ethics Committee (AEC), Khulna University, Bangladesh [Ref: KUAEC-2020/02/02], was issued.

### 2.2. Chemicals

To conduct the analytical and pharmacological test, analytical grade reagents were used, such as DPPH (Sigma, USA), Na_2_CO_3_ (Loba, India), NaNO_2_ (Loba, India), AlCl_3_ (Loba, India), NaOH (Loba, India), H_2_O_2_ (Merck, Germany), Na_2_HPO_4_. 2H_2_O (Loba, India), NaH_2_PO_4_.2H_2_O (Loba, India), FC reagent (Merck, Germany), gallic acid (Sigma Aldrich, USA), quercetin (Merck, Germany), FeCl_3_ (Merck, Germany), PMS (Sigma, USA), NADH (Sigma, USA), NBT (Sigma, USA), and ascorbic acid (Sigma Aldrich, USA). Diclofenac Na and ibuprofen from Square Pharmaceuticals Ltd., Bangladesh, and paracetamol from ACI Pharmaceuticals Ltd., Bangladesh, were procured.

### 2.3. Phytochemical Screening

Qualitative phytochemical screening of the SC extract was carried out according to the method described by Kundu et al. [8]. These tests were conducted to determine the presence of different phytochemical groups.

### 2.4. Test for *In Vitro* Antioxidant Activity

1. Qualitative antioxidative assay

A qualitative antioxidative test of SC extract using the thin-layer chromatography (TLC) technique was done by the method of Sadhu et al. [9]. A small amount of plant extract was diluted in methanol and then spotted on TLC plates precoated with silica gel. After developing the chromatogram by keeping the plates in different solvent systems, those were dried and placed under UV light at both 254 nm and 366 nm to observe the UV active and fluorescent compounds. Finally, 0.02% *w*/*v* DPPH solution in methanol was sprayed on the plates, and the presence of antioxidant components was confirmed by visualizing the yellowish spots.

(2) Quantitative antioxidative assay
  (a) Determination of the content of secondary metabolites
    - Total phenolic content (TPC) assay
    - TPC of the SC extract was measured by using Folin-Ciocalteu (FC) reagent while analytical grade gallic acid was used as the standard [10]. From the calibration curve, TPC was expressed as mg gallic acid equivalent per gram (GAE/gm) of dry extract.
    - Total Flavonoid content (TFC) assay
    - TFC of the SC extract was determined using aluminum chloride colorimetric assay while quercetin was used as standard [10]. From the calibration curve, TFC was expressed as mg quercetin equivalent per gram (QE/gm) of dry extract.
    - Total tannin content (TTC) assay
    - TTC of the SC extract was determined using the FC reagents [10], while gallic acid was used as standard. From the calibration curve, TTC was expressed as mg GAE/gm of dry extract.
  (b) Scavenging of free radicals
    - DPPH free radical scavenging assay
    - DPPH free radicals scavenging of SC extract was carried out by the method of Biswas et al. [11]. Different concentrations of plant sample (16, 32, 64, 128, 512, 1024, and 2048 *μ*g/ml) and ascorbic acid (1, 2, 4, 8, 16, 32, 64, 128, 256, and 512 *μ*g/ml) were prepared, and 0.008% DPPH solution (in methanol) was added to each concentration. Free radical scavenging activity was calculated from the calibration curve of log concentration vs. percent inhibition of DPPH free radical formation. It was expressed as SC_50_ in *μ*g/ml (concentration of sample needed to scavenge 50% radical).
    - Hydrogen peroxide scavenging assay
    - In an aqueous solution, H_2_O_2_ readily dissociates into hydrogen (H^+^) and hydroxyl (OH^−^) radicals [12]. These radicals from H_2_O_2_ were scavenged by the method described by Golder et al. [13] with minor modifications. In this assay, different concentrations of SC extract (12.5, 25, 50, 100, 200, 400, 800, and 1600 *μ*g/ml) and ascorbic acid (1.562, 3.125, 6.25, 12.5, 25, 50, 100, 200, and 400 *μ*g/ml) were prepared, and H_2_O_2_ (40 mM) was added to each concentration. Free radical scavenging activity was calculated from the calibration curve of log concentration vs. percent inhibition of H_2_O_2_ radical formation. It was expressed as SC_50_ in *μ*g/ml.
    - Superoxide radical scavenging assay
    - Superoxide radical was scavenged by the method described by Debnath et al. [14]. In this assay, different concentrations of SC extract (12.5, 25, 50, 100, 200, 400, 8000, and 1600 *μ*g/ml) and ascorbic acid (6.25, 12.5, 25, 50, 100, 200, 400, 8000, and 1600 *μ*g/ml) were prepared. After generating superoxide radical from NBT (312 *μ*M), NADH (936 *μ*M), and PMS (120 *μ*M), those were mixed with the prepared plant solutions. Superoxide radical scavenging activity was calculated from the calibration curve of log concentration vs. percent inhibition of superoxide radical formation. It was expressed as SC_50_ in *μ*g/ml.
  (c) Reducing power assay
  Reducing power of antioxidants may be capable of converting ferric iron to ferrous iron. This process is very beneficial to human health [15]. FeCl_3_ reducing power of SC extract was measured according to the method described by Debnath et al. [16]. Different concentrations of SC extract and ascorbic acid were prepared (12.5, 25, 50, 100, 200, 400, and 800 *μ*g/ml). 0.2 M phosphate buffer, 1% potassium ferricyanide, 10% trichloroacetic acid, and 0.1% FeCl_3_. Reducing ability was calculated from the calibration curve of log concentration vs. percent reduction of FeCl_3_. It was expressed as RC_50_ in *μ*g/ml (concentration of samples required to reduce 50% Fe^3+^).

### 2.5. Screening of Analgesic Activity

(1) Screening of peripheral analgesic activity by acetic acid-induced writhing method
Peripheral analgesic activity of SC extract was tested using the model of acetic acid-induced writhing in mice according to the method described by Debnath et al. [16]. SC extract at 250 and 500 mg/kg and diclofenac Na at 25 mg/kg bw doses were orally administered to different mouse groups. After 30 min, 0.7% *v*/*v* acetic acid was administered intraperitoneally to induce pain or writhing. Then, after 5 min, no. of writhing was counted for the next 15 min for each mouse.
The percentage of writhing inhibition in comparison to the control group was taken as an index of analgesia and was ascertained using the following formula:
  (1) $$\begin{array}{c} \text{Inhibition of writhing }\left(\%\right)=\left[\frac{\left(W_{c}–W_{t}\right)}{W_{c}}\right]\times 100, \end{array}$$
  where *W*_*c*_ is the average number of writhings in the control group and *W*_*t*_ is the average number of writhings in the test group
(2) Evaluation of central analgesic activity by tail immersion method
Central analgesic activity of SC extract was evaluated by the tail immersion method described by Saha et al. with slight modifications [17]. Selected mice were placed in a suitable restrainer keeping the tails spreading out. The lower 5 cm part of the tail was sunk in a beaker of water maintained at 55 ± 0.5°C. That initial reaction time was taken. Then, the SC extract at 250 and 500 mg/kg and tramadol at 10 mg/kg bw doses were orally administered to the test groups [18]. After 1 hr, the reaction time for tail immersion was again recorded. The increase in time was considered an analgesic effect and was calculated by the following equation [19]:
  (2) $$\begin{array}{c} \text{Elongation }\left(\%\right)=\left[\frac{\left(T_{t}–T_{c}\right)}{T_{t}}\right]\times 100, \end{array}$$
  where *T*_*t*_ is the tail immersion time for test group and *T*_*c*_ is the tail immersion time for control group.

### 2.6. Evaluation of Anti-Inflammatory Activity by Formalin-Induced Paw Edema Method

After obtaining a good response from the analgesic test, the anti-inflammatory activity of SC extract was experimented with using the model of formalin-induced paw edema method in mice described by Jahan et al. [10]. SC extract at 250 and 500 mg/kg and ibuprofen at 100 mg/kg bw doses were administered orally to different mouse groups. After 30 min, 0.2% of 0.1 ml formalin solution was injected into the right-back paw of the mice for inducing paw edema. Change in paw size was determined from the paw diameter after and before formalin injection.

(3) $$\begin{array}{c} \text{Inhibition of paw edema or inflammation }\left(\%\right)=\left(\frac{I_{c}–I_{t}}{I_{c}}\right)\times 100, \end{array}$$

where *I*_*c*_ is the inflammation of control group and *I*_*t*_ is the inflammation of test group.

### 2.7. Evaluation of Antipyretic Activity by Brewer's Yeast-Induced Pyrexia Method

The antipyretic effect of SC extract was analyzed by Brewer's yeast-induced hyperthermia in mice modeled by the method described by Subedi et al. [20]. Mice were randomly selected, and the initial rectal temperature was recorded. The selected mice were subcutaneously injected with a 15% *w*/*v* suspension of Brewer's yeast in distilled water at a dose of 10 ml/kg. After 18 hr of injection, the rectal temperature was again recorded. Mice that did not show an increase of a minimum of 0.5°F were excluded from the experiment. Then, those mice were grouped into four groups, where each group consisted of five mice. SC extract at 250 and 500 mg/kg and paracetamol at 150 mg/kg bw doses were administered orally to different mouse groups while mice of the control group were administered with a 1% Tween 80 solution. The rectal temperature of all mice was recorded every hour up to the next 4 hr at regular intervals.

### 2.8. *In Silico* Analysis

Protein preparations: Protein models PDB ID: 5O0X (NOX5), PDB ID: 5KIR (COX 2), and PDB ID: 5C1M (mu-opioid) were selected and downloaded from the protein data bank (https://www.rcsb.org/) to perform molecular docking. Then, protein models were prepared via Discovery Studio 2020 client [21], and at last, energy was minimized using SwissPDB viewer [22] where the grid dimensions were *x* : *y* : *z* = 25.74 : 29.44 : 25, 27.62 : 24.56 : 25, and 24.03 : 23.23 : 25 for 5O0X, 5KIR, and 5C1M, respectively.

Ligand preparation: 3D structures of the standard drugs used in the pharmacological tests, diclofenac Na (CID: 3033), ibuprofen (CID: 3672), paracetamol (CID: 1983), and tramadol (CID: 33741) were downloaded from PubChem (https://pubchem.ncbi.nlm.nih.gov/). We took six antioxidant molecules named as vanillic acid [23], oleanolic acid [24], maslinic acid [25], luteolin [5], myricetin [26], and ellagic acid [27] from the SC extract for in silico analysis as these antioxidant compounds are confirmed to be present in SC fruits by different reports [3–6].

Therefore, these ligands were also downloaded from PubChem (https://pubchem.ncbi.nlm.nih.gov/) [vanillic acid (CID: 8468), oleanolic acid (CID: 10494), maslinic acid (CID: 73659), luteolin (CID: 5280445), myricetin (CID: 5281672), and ellagic acid (CID: 5281855)]. After that, ligand preparation was completed by PyRx [28, 29].

Molecular docking and visualization: site-specific molecular docking analysis was performed in PyRx accumulated with auto dock vina 4.2 [28], and finally, the results were studied in ligplot version 2.2.4 [30].

### 2.9. Statistical Analysis

The experimental data presented here are expressed as mean ± standard deviation (SD). One-way ANOVA test was selected to conduct a statistical comparison of values among the groups (*P* < 0.05 was considered statistically significant) followed by Tukey as a post hoc test by using SPSS (version 25). The graphs were prepared using Graph pad prism software (version 6) [31].

## 3. Results

### 3.1. Phytochemical Test

From the phytochemical assay, SC extract revealed the presence of several types of secondary metabolites such as reducing sugars, tannins, saponins, flavonoids, gums, steroids, glycosides, and terpenoids (Table 1).

### 3.2. Test for *In Vitro* Antioxidant Activity

#### 3.2.1. Qualitative Antioxidant Test

After applying spots on TLC plates and observation under UV light at 254 and 366 nm, the existence of various UV positive and fluorescence active components was detected. After spraying the TLC plates with DPPH solution, the yellow spots indicated the entity of antioxidant compounds in SC extract.

#### 3.2.2. Determination of the Content of Secondary Metabolites

Phenolics, flavonoids, and tannins are mostly common antioxidant compounds found in different plant extracts as secondary metabolites. In our quantitative antioxidant assay, total phenolic, flavonoid, and tannin contents of SC extract were found to be 122 mg GAE/gm, 613 mg QE/gm, and 30 mg GAE/gm, respectively (Table 2 and Figure 3).

#### 3.2.3. Radical Scavenging Activity

To determine the radical scavenging ability of the SC extract, we performed different types of radical scavenging tests. In DPPH free radical scavenging assay, different concentrations of both SC extract and ascorbic acid caused the scavenging of free radicals obtained from DPPH. The calculated SC_50_ values were 87 and 15 *μ*g/ml for SC extract and ascorbic acid, respectively (Table 2 and Figure 4(a)).

In the H_2_O_2_ scavenging assay, SC extract and ascorbic acid scavenged the formed radicals. The calculated SC_50_ values of SC extract and ascorbic acid were 66 and 11 *μ*g/ml, respectively (Table 2 and Figure 4(b)).

In the superoxide radical scavenging assay, different concentrations of both SC extract and ascorbic acid caused the scavenging of the superoxide radicals. With these results, the calculated SC_50_ values of SC extract and ascorbic acid were 347 and 111 *μ*g/ml, respectively. (Tables 2 and Table 3).

#### 3.2.4. Reducing Power Assay

In the reducing power assay, both SC extract and ascorbic acid showed FeCl_3_ reducing ability, and with these results, the RC_50_ values of SC extract and ascorbic acid were 80 and 28 *μ*g/ml, respectively (Table 2 and Figure 4(d)). In this test, the highest absorbance found for the 800 *μ*g/ml solution was 1.296 ± 0.002, whereas that for ascorbic acid was 1.653 ± 0.002.

#### 3.2.5. Evaluation of Peripheral Analgesic Activity by Acetic Acid-induced Writhing Method

In the acetic acid-induced writhing test, SC extract manifested significant writhing inhibition by 20.74% and 39.26% for the doses of 250 and 500 mg/kg bw, respectively. The positive control (diclofenac Na) showed 78.52% writhing inhibition with 25 mg/kg dose (Table 4).

#### 3.2.6. Evaluation of Central Analgesic Activity by Tail Immersion Method

In the tail immersion test, SC extract showed elongation in the tail immersion time up to 22.5% and 37.5% at 250 and 500 mg/kg bw doses, respectively, whereas tramadol at 10 mg/kg bw dose elongated time up to 55.84% (Table 3).

#### 3.2.7. Evaluation of Anti-inflammatory Activity by Formalin-induced Paw Edema Method

In the formalin-induced paw edema test, SC extract showed a significant reduction of edema in the paw of mice within the observing period in a dose-dependent manner (Figure 5).

#### 3.2.8. Evaluation of Antipyretic Activity by Brewer's Yeast-induced Pyrexia Method

In Brewer's yeast-induced pyrexia test, SC extract showed a significant reduction in rectal temperature of mice within the observing period at both the doses of 250 and 500 mg/kg (Figure 6).

#### 3.2.9. *In Silico* Analysis

From the above-mentioned *in vitro* antioxidative tests, we found that SC extract possesses good antioxidant content. Therefore, we went to conduct the *in silico* analysis for the antioxidant molecules reported being present in this extract (Figure 4). Here, ellagic acid revealed the highest binding affinity (–10.9 kcal/mol) for *Cylindrospermum stagnale* NADPH-oxidase 5 (NOX5) (PDB ID: 5O0X), whereas the binding affinity of the standard ascorbic acid was –5.3 kcal/mol (Table 5).

SC extract exhibited significant analgesic (both central and peripheral), anti-inflammatory, and antipyretic effects. So, we went to execute an *in silico* analysis for those properties using antioxidant molecules as plant-derived antioxidants like polyphenolic compounds, flavonoids, tannins, and terpenoids have been reported for expressing those effects [32]. In the case of peripheral analgesic, anti-inflammatory, and antipyretic properties, luteolin revealed –9.6 kcal/mol as the highest binding affinity, whereas the standard drugs diclofenac Na, ibuprofen, and paracetamol exhibited binding affinity of –7.1, –7.3, and –6.1 kcal/mol, respectively, against the COX 2 enzyme (Table 6). For the central analgesic property, ellagic acid presented the highest binding affinity of –8.6 kcal/mol, and that for the standard drug tramadol was –6.4 kcal/mol against mu (*μ*) opioid receptor (Table 7).

## 4. Discussion

Nature has always blessed mankind with its numerous medicinal plants to protect against many diseases and sufferings. Most plants are a monstrous storehouse of various phytochemicals which are divided into primary and secondary metabolites. Secondary metabolites are the main therapeutically important compounds as they exhibit diverse pharmacological activities which are beneficial to both the plant itself and humans. From the very ancient period to the modern age, man has always sought newer drugs from these blessings of nature [33]. Our phytochemical investigation revealed that the SC extract is enriched with different types of phytochemicals, and these might be very helpful to elicit different biological responses.

Due to the presence of different types of important phytochemical groups as secondary metabolites like flavonoids, polyphenolics, tannins, and vitamins, mangrove plants are a great source of antioxidant compounds [34]. Among these types, phenols, flavonoids, and tannins are the most common and abundant types of antioxidant compounds found in plant species. In humans, many phenolic compounds may be capable of preventing the risk of developing many chronic diseases like cancer, diabetes, and cardiovascular disease. Tannins are also capable of reducing lipid peroxidation and DNA mutations [35], and flavonoids showed antispasmodic, antiallergic, and anti-inflammatory activities as well as protective effects on vascular and hepatic disorders [36].

Free radicals are regularly produced in our bodies. In our normal physiological process, lipid peroxidation happens, and it then stimulates oxidation of sulfhydryl groups, deformation of protein, and segmentation of DNA bases, and ultimately, these cause different serious diseases like inflammation, cardiovascular and respiratory disorders, cancer, atherosclerosis, diabetes, and neurological disorders [31, 37]. DPPH is a common stable radical that can easily receive an electron or proton from antioxidant molecules and be converted into a yellowish color [38]. H_2_O_2_ is also a strong oxidative agent which generates hydroxyl radicals (OH) in an aqueous solution. On the other hand, superoxide radical is harmful to cellular components. As a precursor of reactive oxygen species, it damages tissues and cells and thus causes various diseases [39]. Antioxidants can neutralize the formed ROS [40, 41].

Antioxidants not only serve as free radical scavengers but also act as reducing agents. The reducing ability of the antioxidants is also beneficial for our health. SC extract showed a good reducing ability in reducing FeCl_3_. From the results of different radical scavenging tests and reducing power assays, we can summarize that SC fruits might be a very potent source of antioxidants that might be used to neutralize free radicals and thus may protect our body from the accompanying diseases.

Algesia (G. *algesis*) or pain is always an unpleasant sensation. It is usually provoked by external or internal obnoxious stimuli. These tend to release arachidonic acid from the phospholipids of the affected tissues. As a result, the secretion of many intracellular components arises. The secreted prostacyclin (PGI_2_), PGE_2_ and PGF_2*α*_, cytokines, and leukotrienes have been held responsible for the sensation of pain [42]. The acetic acid-induced writhing method in mice is a widely used test for screening the peripheral analgesic effect. Intraperitoneal administration of acetic acid induces different endogenous pain mediators that sensitize pain nerve terminals [43]. In this test, SC extract expressed significant writhing impulse inhibition at both 250 mg/kg and 500 mg/kg doses, and the observed responses were found in a dose-dependent manner.

The brain and spinal cord play a crucial role in the central pain mechanism. The dorsal part of the spinal cord is enriched with substances like prostaglandins, somatostatins, bradykinins, and many other inhibitory pain-targeting biomolecules. To measure the central analgesic effect, tail-flick and tail immersion models are well-established methods [17]. Central analgesic drugs like opioids, tramadol, and dextropropoxyphene elicit analgesic responses through binding to opioid receptors. In our experiment, SC extract showed a central analgesic effect by elongating the tail immersion time in both doses.

Like pain, inflammation is another type of normal cellular response of living tissues to injury or other external stimuli. It is another body defense system to eliminate or limit the spread of the pathogenic injurious agent. To measure the anti-inflammatory activity, formalin-induced paw edema is a widespread widely accepted test. Intraplantar injection of formalin solution produces the release of inflammatory mediators like prostaglandins, bradykinins, and serotonin [44]. Ibuprofen, as with other conventional NSAIDs (nonsteroidal anti-inflammatory drugs), also reduces the synthesis of pain and the associated inflammatory mediators [45]. In the anti-inflammatory test, SC extract expressed a significant dose-dependent reduction in paw edema size in mice within the observing period.

Inflammation, pain, and pyrexia underlie several pathological conditions associated with different types of mediators which are produced by similar mechanisms [46]. Pyrexia or hyperthermia is usually generated as an associated impact of cellular infection, tissue damage, malignancy, graft rejection, and/or other pathological conditions. Normally, the affected tissues initiate the excess formation of different proinflammatory mediators (cytokines like interleukin-1*β*, interleukin-1*α*, and TNF-*α*). These trigger the increase in the synthesis of prostaglandin E_2_ (PGE_2_) and PGI_2_ near the hypothalamus zone and induce the hypothalamus to raise the body temperature [47]. Brewer's yeast-induced pyrexia is a reliable method that is used to assess the antipyretic effect of any sample. Different proteins presented in yeast are linked to fever via the synthesis of different fever mediatory cytokines, interleukins, and prostaglandins. Antipyretic drugs like paracetamol and many other conventional NSAIDs generally affect the cyclooxygenase (COX) pathway and reduce the production of fever-generating mediators and thus normalize the elevated body temperature [20]. In the antipyretic test, SC extract showed a good antipyretic effect by lowering the rectal temperature of mice over the observing period. Therefore, we can suggest that SC extract might have an antipyretic property through the mechanism discussed above.

Although there are sufficient analgesic, anti-inflammatory, and antipyretic agents in the drug market, the most prevalent side effects are gastrointestinal damage, peptic ulcer, bleeding, and renal and liver damage. Most synthetic COX inhibitors are highly selective to hepatic, renal, cardiac, and glial cells, and thus, they cause unwanted adverse effects. On the other hand, natural COX inhibitors are safe for use as they lack the high selectivity to the above cells [47]. With the increasing cost of synthetic drugs, most people, especially in poor and developing countries, rely on natural compounds, and those are also quite free from adverse effects. Foods rich in antioxidant contents have been used for many decades to boost our immune system so that we can protect ourselves from many free radical-mediated diseases. There lies an inverse relationship between the consumption of dietary antioxidants and illness. Most polyphenolic compounds like flavonoids and tannins act by blocking the arachidonic acid metabolic pathway, and thus, they inhibit the enzymes involved in inflammation and other mediators that are responsible for pain perception, inflammatory responses, and fever [48, 49]. Besides polyphenolics, flavonoids, terpenoids, and alkaloids are also reported for expressing analgesic and anti-inflammatory properties [32].

From the antioxidative tests, we have found that SC extract is enriched in antioxidant components, and we also observed good analgesic, anti-inflammatory, and antipyretic responses from the *in vivo* tests. As it is already mentioned that antioxidants have significant roles in treating inflammation and associated diseases, so it is supposed that antioxidant molecules reported in this plant such as vanillic acid (a phenolic compound) [50], oleanolic acid (a triterpenoid) [51], maslinic acid (a triterpenoid) [52], luteolin (a flavonoid) [53], myricetin (a polyphenolic compound) [54], and ellagic acid (a polyphenolic compound) [55] might be responsible for the mentioned pharmacological effects (Figure 7). Therefore, we aimed to conduct the *in silico* study of these antioxidant compounds to determine the better binding affinities with related receptors.

NADPH oxidase (NOX5) is a vital enzyme that is responsible for the generation of many reactive oxygen species in the biological system. 5O0X is a receptor of NOX5, and it was already reported by Islam et al. for *in silico* analysis of antioxidant potentials [56]. Considering this fact, we also took that 5O0X receptor to conduct *in silico* analysis of antioxidant molecules present in SC extract along with ascorbic acid, a well-known antioxidant. From our analysis, the highest binding affinity was found for ellagic acid (–10.9 kcal/mol), whereas the binding affinity of ascorbic acid was –5.3 kcal/mol. Luteolin and myricetin were also found to have notable binding affinities (Table 5). There were some common binding regions of the antioxidant molecules along with ascorbic acid (Figure 8). Most of the binding amino acid residues are the same, for example, Ile538, Phe461, Trp695, Pro460, Arg478, Thr462, His476, Thr541, and Ile477 (Figure 9, Table 5).

To conduct *in silico* analysis of the antioxidant molecules for peripheral analgesic, anti-inflammatory, and antipyretic effects, we took 5KIR as a protein of COX enzyme of the human body as it is already reported by Emon et al. [57]. From our analysis, the highest binding affinity was found for luteolin (–9.6 kcal/mol), which was found higher than standard drugs (binding affinities of diclofenac Na, ibuprofen, and paracetamol were –7.1, –7.3, and –6.1 kcal/mol, respectively). Along with this, oleanolic acid, myricetin, and ellagic acid were also found notable binding affinities to the 5KIR protein (Table 6).  Figure 10 indicates the binding of luteolin and the standard drugs in a quite similar region, and most of the binding amino acid residues are the same, namely, Val349, Ser353, Trp387, Leu352, Phe518, Tyr355, Val523, His90, Ile517, Ala516, and Gln192 (Figure 11, Table 6). Therefore, it could be assumed that luteolin plays a major role in exerting peripheral analgesic, anti-inflammatory, and antipyretic activities of SC extract by inhibiting COX enzymes.

Different mu (*μ*) receptors in our brain are responsible for central pain sensation. In a previous article, Aljohani et al. conducted an *in silico* analysis of the central analgesic activity by taking the 5C1M protein of *μ* receptors [58]. We also took that 5C1M protein, and it was docked with the above-mentioned ligands and the standard drug tramadol. We found that the binding affinity of ellagic acid was –8.6 kcal/mol, which was better than that of tramadol –6.4 kcal/mol. Luteolin and myricetin also showed better binding affinities (Table 7). We also found that tramadol and ellagic acid are bound in the same binding region (Figure 12), and most of the binding amino acid residues are the same, namely, Ile296, Val 300, Tyr326, His297, Tyr148, and Asp147 (Figure 13, Table 7). Thus, it can be concluded that ellagic acid might be responsible for exerting the central analgesic activity of the plant extract by the inhibition of the *μ* receptor.

## 5. Conclusion

Our present study was conducted on the fruits of *S. caseolaris* to investigate its antioxidative, analgesic, anti-inflammatory, and antipyretic properties along with *in silico* analysis. From our observation, we can conclude that these fruits are highly enriched in antioxidative compounds, and they can serve as a food supplement to protect our body from different oxidative disorders and associated diseases. This extract also showed a good response in analgesic, anti-inflammatory, and antipyretic tests, and those responses were further confirmed by molecular docking analysis in which ellagic acid and luteolin were found to be the most active components responsible for the effects. The results also justify its traditional usage in folklore medicine. Based on our findings, we can suggest *S. caseolaris* fruits might be a potential source of medicinal components in alleviating inflammation. These preliminary results might help natural product scientists to find out better lead molecules from this plant in the future, and those will surely contribute to the modern medicine system.

## Figures and Tables

**Figure 1:** Photo of *S. caseolaris* fruits.

**Figure 2:** Schematic diagram of the experimental program.

**Figure 3:** Calibration curve of (a) gallic acid for determining total phenolic content, (b) quercetin for determining total flavonoid content, and (c) gallic acid for determining total tannin content.

**Figure 4:** (a) % scavenging of DPPH free radical vs. log concentration of *S. caseolaris* extract and ascorbic acid, (b) % scavenging of H_2_O_2_ vs. log concentration of *S. caseolaris* extract and ascorbic acid, (c) % scavenging of superoxide radical vs. log concentration of *S. caseolaris* extract and ascorbic acid, and (d) % reducing of FeCl_3_ vs. log concentration of *S. caseolaris* extract and ascorbic acid.

**Figure 5:** Comparison of paw thickness (mm) at different times for control, standard and *S. caseolaris* extract in the formalin-induced paw edema method.

**Figure 6:** Comparison of rectal temperature (°F) at different times for control, standard, and *S. caseolaris* extract in Brewer's yeast-induced pyrexia method.

**Figure 7:** Chemical structures of (a) vanillic acid, (b) oleanolic acid, (c) maslinic acid, (d) luteolin, (e) myricetin, and (f) ellagic acid.

**Figure 8:** Binding of ellagic acid (red) and ascorbic acid (green) with NOX5 protein.

**Figure 9:** 2D interactions of amino acids with (a) ellagic acid and (b) ascorbic acid.

**Figure 10:** Binding of diclofenac Na (red), ibuprofen (green), paracetamol (blue), and luteolin (yellow) with COX 2 receptor.

**Figure 11:** 2D interactions of amino acids with (a) diclofenac Na, (b) ibuprofen, (c) paracetamol, and (d) luteolin.

**Figure 12:** Binding of tramadol (green) and ellagic acid (red) with 5C1M protein of mu receptor.

**Figure 13:** 2D interactions of amino acids with (a) tramadol and (b) ellagic acid.

**Table 1:** Presence or absence of phytochemical groups in *S. caseolaris* extract.

Phytochemical groups	SC extract
+	Reducing sugars
+	Tannins
+	Flavonoids
+	Saponins
+	Gums
+	Steroids
-	Alkaloids
+	Glycosides
-	Xanthoproteins
+	Terpenoids
-	Acidic compounds

“+” indicates the presence, and “-” indicates the absence.

**Table 2:** Total content of secondary metabolites and approximate SC_50_ values of different radicals scavenging assays and RC_50_ of reducing power assay of *S. caseolaris* extract.

Sample	TPC (mg GAE/g)	TFC (mg QE/g)	TTC (mg GAE/g)	DRSA (SC_50_*μ*g/ml)	HPSA (SC_50_*μ*g/ml)	SRSA (SC_50_*μ*g/ml)	RPA (RC_50_*μ*g/ml)
SC extract	122	613	30	87	66	347	80
Ascorbic acid	—	—	—	15	11	114	28

TPC: total phenolic content; TFC: total flavonoid content; TTC: total tannin content; DRSA: DPPH radical scavenging activity; HPSA: hydrogen peroxide scavenging activity; SRSA: superoxide radical scavenging activity; RPA: reducing power assay.

**Table 3:** Effects of *S. caseolaris* extract on tail withdrawal reflexes in tail immersion method in mice.

Treatment group	Dose (mg/kg)	Before treatment	After treatment	% inhibition of pain
Negative control	—	5.02 ± 0.16	5.1 ± 0.14^*θ*▲∆^	—
Standard (tramadol)	10	5.26 ± 0.31	11.55 ± 0.44^∗^^▲∆^	55.84
SC extract	250	5.05 ± 0.23	6.58 ± 0.57^∗^^*θ*∆^	22.05
SC extract	500	5.02 ± 0.29	8.16 ± 0.65^∗^^*θ*▲^	37.5

Data are means of five replicates ± SD; ^∗^*P* < 0.05 vs. control (Dunnett's *t* test); *^*θ*^P* < 0.05 vs. tramadol 10 mg/kg; ^▲^*P* < 0.05 vs. SC extract 250 mg/kg; ^∆^*P* < 0.05 vs. SC extract 500 mg/kg (pair-wise comparison by post hoc Tukey test).

**Table 4:** Effects of *S. caseolaris* extract on acetic acid-induced writhing in mice.

Treatment group	Dose (mg/kg)	Mean writhing	% inhibition of writhing
Negative control	—	27 ± 2.00^*θ*▲∆^	—
Standard (diclofenac Na)	25	5.8 ± 0.84^∗^^▲∆^	78.52
SC extract	250	21.4 ± 1.95^∗^^*θ*∆^	20.74
SC extract	500	16.4 ± 2.30^∗^^*θ*▲^	39.26

Data are means of five replicates ± SD; ^∗^*P* < 0.05 vs. control (Dunnett's *t* test); *^*θ*^P* < 0.05 vs. diclofenac Na 25 mg/kg; ^▲^*P* < 0.05 vs. SC extract 250 mg/kg; ^∆^*P* < 0.05 vs. SC extract 500 mg/kg (pair-wise comparison by post hoc Tukey test).

**Table 5:** Binding characteristics of ligands against NOX5 proteins.

Ligands	Protein	Binding affinity (kcal/mol)	Interacting amino acids
Ascorbic acid	NOX5	–5.3	Ile538, Phe461, Trp695, Pro460, Thr462, His476, Thr541
Vanillic acid		–6.4	Thr462, Thr541, Arg478, His476, Ile538, Phe461, Trp695, Pro460, Ile477
Oleanolic acid		–7.7	Ile538, Arg478, Phe461, Pro460, Pro694, Val480, Thr484, Trp695
Maslinic acid		–7.8	Ile538, Trp695, Phe461, Pro460, Pro694, Arg478, Val480, Thr484
**Luteolin**		–**9.4**	Arg478, His476, Thr462, Ile538, Phe461, Ile477, Tyr 445, Pro460, Trp695, Thr484, Val480
**Myricetin**		–**8.9**	Thr462, His476, Arg478, His459, Ile477, Ile538, Thr541, Phe461, Pro460, Trp695, Val480, Thr484
**Ellagic acid**		–**10.9**	Arg478, Thr541, Thr462, Ile538, Trp695, Pro460, Tyr 445, Phe461, His476

Compounds marked bold showed the best binding affinities.

**Table 6:** Binding characteristics of ligands against COX 2.

Ligands	Protein	Binding affinity (kcal/mol)	Interacting amino acids
Diclofenac Na	5KIR	–7.1	Phe518, Val523, Met522, Leu352, Trp387, Ser530, Tyr385, Ala527, Val349, Ser353, Arg120, Tyr355
Ibuprofen		–7.3	Tyr355, His90, Phe518, Val523, Ala527, Ser530, Tyr385, Gly526, Trp387, Val349, Ser353, Leu352, Arg513
Rofecoxib		–9.7	Phe518, Ile517, Ala516, Arg513, His90, Leu352, Trp387, Met522, Ala527, Gly526, Val349, Val523, Ser353, Gln192, Tyr355
Vanillic acid		–6.3	Leu390, Ala199, Trp387, Glu203, Ala202, Thr206, His207, His388, Tyr385, His386, Leu391
Oleanolic acid		–**8.1**	Gln192, Gly354, His351, Asn350, Asp347, Ile564, Tyr355, His356
Maslinic acid		–7.7	Tyr355, His356, Gln192, His351, Phe580, Gly354, Asp347, Ser579, Ile564
Luteolin		–**9.6**	Tyr385, Ser530, Val349, Ser353, Trp387, Leu352, Phe518, Tyr355, Val523, His90, Ile517, Ala516, Gln192
Myricetin		–**8.8**	Tyr385, Ala527, Gly526, Val349, His90, Ser353, Tyr355, Gln192, Val523, Ile517, Phe518, Leu352, Ala516, Trp387, Leu384, Ser530,
Ellagic acid		–**8.3**	Phe580, Ser581, His351, Asp347, Tyr355, Asn350, Ser579

Compounds marked bold showed the best binding affinities.

**Table 7:** Binding characteristics of ligands against mu (*μ*) opioid receptor.

Ligands	Protein	Binding affinity (kcal/mol)	Interacting amino acids
Tramadol	5C1M	–6.4	His54, Gln124, Met151, Tyr326, Trp293, Asp147, Tyr148, Ile296, Val236, Val300
Vanillic acid		–5.4	Val300, Ile296, Val236, His297, Trp293, Ile322, Tyr326, Asp147, Met151, Val236
Oleanolic acid		–6.4	Ile146, Trp192, Leu116, Tyr149, Leu112, Asn109, Thr153, Asn150
Maslinic acid		–6.7	Asn150, Tyr149, Trp192, Asn109, Phe108, Leu112, Leu116, Lle146
Luteolin		**–7.9**	Leu232, Lys233, Val300, Val236, Tyr148, Asp147, Ile322, Tyr326, Gln124, Ile296, His297
Myricetin		**–7.6**	His297, Ile296, Glu124, Ile322, His54, Ile144, Asp147, Tyr148, Val236, Val300
Ellagic acid		**–8.6**	His297, Val300, Ile296, Tyr148, His54, Asp147, Gln124, Tyr326

Compounds marked bold showed the best binding affinities.

## Data Availability

The experimental data of this manuscript are preserved on our computer, and those will be available upon request.

## Abbreviations

SC: *Sonneratia caseolaris*
mg: Milligram
ml: Milliliter
*μ*g: Microgram
kg: Kilogram
*μ*l: Microliter
DPPH: 2,2-Diphenyl-1-picryl hydrazyl
PMS: Phenazine methosulphate
NBT: Nitroblue tetrazolium
NADH: Nicotinamide adenine dinucleotide
bw: Body weight
NST: National Science and Technology
AEC: Animal Ethics Committee
ANOVA: Analysis of variance.
